The article "The Influence of Intraoperative Ultrasound Monitoring on the Risk of Recurrence and Reoperation in Patients with Hysteromyomectomy" was published in 2022. Journal: Contrast Media Mol Imaging.

# The Influence of Intraoperative Ultrasound Monitoring on the Risk of Recurrence and Reoperation in Patients with Hysteromyomectomy

**DOI:** 10.1155/2022/4366840

**Published:** 2022-06-09

**Authors:** Sanmei Yu, Yanni Xiang

**Affiliations:** Department of Ultrasound, Taizhou First People's Hospital, Taizhou 318020, Zhejiang, China

## Abstract

In recent years, with the continuous development and application of minimally invasive methods in China, laparoscopic myomectomy has become the primary method for clinical treatment of uterine fibroids. There is also a high risk of recurrence and reoperation after endoscopic myomectomy. Intraoperative use of ultrasound for auxiliary examination can provide medical staff with spatial information and position information of fibroids and help medical staff to accurately locate the surgical incision. The aim is to investigate the effect of intraoperative ultrasound monitoring on the risk of postoperative recurrence and reoperation in patients undergoing myomectomy. This study retrospectively collected 80 patients who underwent laparoscopic myomectomy in the gynecology department of our hospital from January 2020 to January 2022. According to the different treatment methods, they were divided into a study group and a control group (both *n* = 40). The control group underwent preoperative ultrasonography and then underwent myomectomy, while the study group underwent both preoperative and intraoperative ultrasonography before undergoing hysterectomy. Myomectomy: all the enrolled patients were followed up by ultrasound after surgery and followed up for 1 year (recheck ultrasound every 3 months). The indicators, postoperative complications, postoperative average diameter of uterine fibroids, postoperative residual rate of uterine fibroids, postoperative recurrence, and reoperation were compared between the two groups. Intraoperative ultrasound monitoring has a significant effect on patients undergoing myomectomy, which can effectively reduce the residual rate of fibroids, completely remove small and deep fibroids, and reduce complications, postoperative recurrence, and reoperation risks. It has good clinical application value.

## 1. Introduction

Uterine fibroids are common benign tumors of the female reproductive system, mostly in women of childbearing age, with an incidence of up to 40% [1]. It is mainly caused by the proliferation of smooth muscle cells, formed by fibrous connective tissue, and, can cause irregular vaginal bleeding in female patients, menorrhagia, pelvic pain, frequent urination, constipation, abortion, and infertility and other symptoms. According to data, about 20% to 50% of patients with symptomatic uterine fibroids and 53.7% of patients with symptoms think that the symptoms caused by uterine fibroids have a serious negative impact on their normal work and family happiness [2, 3]. With the continuous progress and application of minimally invasive methods in China, laparoscopic myomectomy has become the primary method for clinical treatment of uterine fibroids due to its advantages of small incision, light pain, and quick postoperative recovery [4]. However, the risk of recurrence and reoperation after laparoscopic myomectomy is also high because the minimal uterine fibroid residue cannot be directly touched during surgery [5]. Some studies have found that ultrasonic monitoring during laparoscopic myomectomy can effectively reduce intraoperative residual and control the recurrence rate without increasing the incidence of postoperative complications [6]. However, there are few reports about the effect of intraoperative ultrasound monitoring on postoperative recurrence and reoperation risk of patients undergoing hysteromyomectomy. Therefore, in this study, this study selected 80 patients who underwent transabdominal myomectomy as the research subjects and explored the influence of intraoperative ultrasound monitoring on postoperative recurrence and reoperation risk of patients undergoing myomectomy.

The article "The Influence of Intraoperative Ultrasound Monitoring on the Risk of Recurrence and Reoperation in Patients with Hysteromyomectomy" was published in 2022. Journal: Contrast Media Mol Imaging.

## 2. Data and Methods

### 2.1. Technical Route

The technical route is shown in Figure 1.

### 2.2. General Information

Eighty patients who underwent laparoscopic myomectomy in our department of gynecology from January 2020 to January 2022 were retrospectively collected. Inclusion criteria: ① patients who meet the diagnostic criteria for uterine fibroids [7] and who were confirmed to have multiple uterine fibroids by clinical examination and surgery after admission; ② all underwent laparoscopic myomectomy; ③ age ≤45 years old and had fertility; ④ clinical symptoms such as heavy menstrual flow, excessive diameter of uterine fibroids, and rapid growth that affect life; ⑤ the patient gave informed consent, actively cooperated with treatment, and agreed to follow-up after surgery. Exclusion criteria: ① with malignant lesions of uterine fibroids; ② with contraindications to laparoscopic surgery; ③ combined with loss of important organ function (such as liver, kidney, and heart) and coagulation dysfunction; ④ those lost to follow-up. The included patients were divided into study group and control group according to different treatment methods (all *n* = 40). Comparison of baseline data between the two groups (*P* > 0.05) (see Table 1).

### 2.3. Methods

All patients routinely completed all preoperative preparations after admission.

The control group underwent laparoscopic myomectomy. All the patients in the group underwent surgical treatment 3 to 7 days after the menstrual period was over. The bladder stones were taken, and general anesthesia was performed. The umbilicus was used as the first puncture hole (10 mm), the reverse McBlanc's point was used as the second puncture hole (10 mm), and the McBlanc's point was used as the third puncture hole (6 mm). Link laparoscopic (German STORZ company) equipment is used to detect and observe the number, diameter, and location of uterine fibroids in patients; to diagnose whether the patient has symptoms such as pelvic adhesions; and to inject vasopressin 6∼12U. The myometrium was incised horizontally to fully expose the uterine fibroids, and then removed, and the uterus was sutured after removal. The uterus was explored by laparoscopy. After there was no residual uterine fibroids, 0.9% sodium chloride solution was used to slowly rinse the uterus. If there was no abnormality, the trocar was removed, the puncture hole was closed, and the dressing was applied.

The article "The Influence of Intraoperative Ultrasound Monitoring on the Risk of Recurrence and Reoperation in Patients with Hysteromyomectomy" was published in 2022. Journal: Contrast Media Mol Imaging.

In the study group, on the basis of the control group, intraoperative ultrasound guidance was added. Ultrasound diagnostic instrument (Siemens OMNI-3 type) was used to monitor patients with intracavitary dynamic ultrasound. The probe frequency was 5–8 MHz, and the rotatable range was 220°. During the operation, the position and depth of the uterine incision were selected under the guidance of ultrasound. If the ultrasound image showed the existence of residual uterine fibroids, the fibroids were located by laparoscopic guide rods, and then the myometrium was incised under the guidance of ultrasound until the fibroids were exposed and completely removed immediately. After the removal is completed, the uterus is sutured. The uterus was explored by laparoscopy. After there was no residual uterine fibroids, 0.9% sodium chloride solution was used to slowly rinse the uterus. If there was no abnormality, the trocar was removed, the puncture hole was closed, and the dressing was applied. Both groups were followed up for 1 year after operation.

### 2.4. Observation Indicators

① Intraoperative indicators (including the amount of bleeding during the operation, operation time, postoperative exhaust time, and hospitalization time) were observed and recorded in 2 groups. ② The incidence of postoperative complications (including disc hematoma, ureteral injury, and vascular nerve injury) was recorded in the two groups. ③ The presence of residual uterine fibroids was determined by intracavitary color Doppler ultrasonography within 3 weeks after surgery. Diagnostic criteria [8]: postoperative ultrasonography showed solid hypoechoic nodules with diameter ≥1.0 cm and clear capsule. Patients were asked to go to the hospital for re-examination 3, 6, and 12 months after surgery. The patients with uterine fibroids with diameter ≥1.0 cm or fibroids with diameter <1 cm and enlargement trend were determined as fibroid recurrence after 3 months of intravascular color Doppler ultrasound. Average postoperative uterine fibroid diameter, uterine fibroid residue, and recurrence were recorded in 2 groups.

The article "The Influence of Intraoperative Ultrasound Monitoring on the Risk of Recurrence and Reoperation in Patients with Hysteromyomectomy" was published in 2022. Journal: Contrast Media Mol Imaging.

### 2.5. Data Analysis Method

SPSS 25.0 statistical software was used for data processing in this study. Measurement data (in accordance with normal distribution) were expressed as ($\bar{x}$ ± *s*) and used the *t*-test; count data were described as rate (%) and used the *χ*^2^ test. The difference was statistically significant with *P* < 0.05.

## 3. The Results

### 3.1. Comparison of Surgical Indicators between the Two Groups

There were no differences in surgical indexes (the amount of bleeding during the operation, operation time, postoperative exhaust time, and hospitalization time) between the two groups (*P* > 0.05) (Table 2).

### 3.2. Comparison of Two Groups of Complication Rate

The incidence of complications in the study group and the control group were 5.00% and 22.50%, respectively, and the comparison was statistically significant (*P* < 0.05) (Table 3).

### 3.3. Comparison of Average Postoperative Uterine Fibroid Diameter between the Two Groups

After surgery, the mean diameter of uterine fibroids in the study group was 0.85 ± 0.24 cm lower than that in the control group (1.39 ± 0.61 cm) (*P* < 0.05) (Figure 2).

### 3.4. Postoperative Ultrasound Examination of Residual Uterine Fibroids in the Two Groups

In the study group, there were 2 cases (5.00%) with uterine muscle residue and 2 fibroids residue in postoperative ultrasound examination. In the control group, 15 cases (37.50%) had residual uterine muscle and 17 fibroids. Compared with the control group, the residual rate of uterine fibroids in the study group was lower (*P* < 0.05) (Figure 3).

### 3.5. Comparison of the Risk of Postoperative Ultrasound Uterine Fibroids Recurrence and Reoperation between the Two Groups

Both groups were followed up for 1 year after operation, and the recurrence rate of uterine fibroids in the two groups was compared from 3 to 6 months after surgery (*P* > 0.05). Comparison of recurrence rate of uterine fibroids between the two groups 6∼12 months after operation (*P* < 0.05). The total recurrence rate of postoperative uterine fibroids in the study group and the control group was 7.50% and 27.50%, respectively. The patients with postoperative recurrence in the two groups all required reoperation, compared between the two groups (*P* < 0.05) as shown in Table 4 and Figure 4.

The article "The Influence of Intraoperative Ultrasound Monitoring on the Risk of Recurrence and Reoperation in Patients with Hysteromyomectomy" was published in 2022. Journal: Contrast Media Mol Imaging.

## 4. Discussion

Uterine fibroids are benign reproductive system tumors mainly dependent on estrogen and progesterone, so the incidence and recurrence rate of women in reproductive period are higher. In order to preserve the fertility function of patients, myomectomy is often used in clinical treatment, including traditional laparotomy and laparoscopic surgery. However, compared with traditional open surgery, laparoscopic myomectomy cannot intuitively touch the uterus and bilateral appendage, and the indirect surgical field also has an impact on the judgment of the presence of uterine fibroid residue [9, 10]. Because uterine fibroids can not be removed clean easy to cause recurrence, causing great psychological burden to patients. Foreign studies have reported that short-term postoperative recurrence rate is as high as 20%∼30%, among which intraoperative fibroid residue is the main cause of recurrence, which can increase the risk of reoperation [11, 12]. Ultrasound is the most sensitive method for the detection of uterine fibroids, which can better display the size, location, and echo of uterine fibroids, and has the characteristics such as noninvasive, simple operation, and strong repeatability. The combination of intraoperative ultrasound and laparoscopy can reduce the risk of fibroid residue. Intraoperative ultrasound monitoring is the combination of ultrasound technology and laparoscopic instruments. The ultrasonic probe enters through the puncture hole and directly contacts the surface of the uterus for scanning and obtains the image of the lesion, so that the operator can obtain information such as the location of the lesion and the relationship between the lesion and its adjacent [13]. Currently, Qinggan Huoxue Recipe and laparoscopic ultrasound are more commonly used in clinical treatment of liver diseases, and the clinical efficacy is good [14, 15]. In terms of gynecology, studies have found that transvaginal ultrasound in laparoscopic surgery can find small fibroids that cannot be detected by the naked eye and remove them, which can minimize fibroid residue and reduce the recurrence rate [16]. Other studies suggest that transvaginal ultrasound plays a greater role in adjuvant treatment of laparoscopic multiple uterine fibroids, which can reduce the residual rate of postoperative uterine fibroids and the 1-year recurrence rate, and the prognosis of patients is good [17]. In addition, it has been reported that laparoscopic ultrasound can detect adenomyosis not detected by preoperative ultrasound [18].

## 5. Results

Although the average operation time was longer in the study group, there was no difference in the surgical indicators (the amount of bleeding during the operation, operation time, postoperative exhaust time, and hospitalization time) between the study group and the control group, indicating that although intraoperative ultrasound-guided laparoscopic myomectomy increases the patient's operation time, it does not affect the safety of the operation, and the patient's postoperative rehabilitation process has no direct impact. The reasons may be as follows: the abdominal incision is smaller during laparoscopic myomectomy, and the postoperative suture pain is less, so the patient's intraoperative blood loss, postoperative exhaust time, and other indicators are lower, while laparoscopic myomectomy is performed. Intraoperative ultrasound monitoring has more monitoring steps and can directly observe the blood flow of patients to guide myomectomy, thereby increasing the operation time, but it does not reduce the efficiency of intraoperative operations [19]. Therefore, there was no significant difference between the two groups of surgical indicators.

The article "The Influence of Intraoperative Ultrasound Monitoring on the Risk of Recurrence and Reoperation in Patients with Hysteromyomectomy" was published in 2022. Journal: Contrast Media Mol Imaging.

In this study, both groups were followed up for 1 year after operation. The results showed that, for the control group, the average postoperative uterine fibroid diameter, uterine fibroid residual rate, uterine fibroid recurrence rate, and reoperation rate were smaller in the study group, suggesting that intraoperative ultrasound-guided laparoscopic myomectomy is effective. Reduce residual fibroids and reduce the risk of postoperative recurrence. The reason for the analysis may be that the problem of omission of deep fibroids between the nonprotruding uterine surface muscle walls can be effectively avoided during surgery under the guidance of intraoperative ultrasound. The size and location of uterine fibroids are determined through blood flow signal analysis, and accurate positioning is carried out to guide the operation. In addition, intraoperative ultrasound monitoring can directly scan the organs, directly discovering problems not found by preoperative ultrasound, improving the diagnostic accuracy, thereby reducing the residual probability and recurrence rate. Pelvic hematoma, ureteral injury, and vascular and nerve injury are common complications after myomectomy, which may occur because some fibroids are close to the endometrium and easily penetrate the uterine cavity or uterine cavity during removal [20, 21]. The results of this study found that the incidence of complications in the control group was 22.50%, while that in the study group was 5.00% (*P* < 0.05). These results suggest that ultrasound monitoring during abdominal mirror myomectomy can effectively reduce complications. The reason for the analysis may be the use of intraoperative ultrasound to determine the spatial position and adjacent relationship of fibroids and to increase the accuracy of the doctor's operation, thereby reducing the incidence of postoperative complications.

The article "The Influence of Intraoperative Ultrasound Monitoring on the Risk of Recurrence and Reoperation in Patients with Hysteromyomectomy" was published in 2022. Journal: Contrast Media Mol Imaging.

## 6. Strengths and Limitations

In this study, the clinical data of 80 patients undergoing transabdominal myomectomy were used to investigate the effect of intraoperative ultrasound monitoring on the risk of postoperative recurrence and reoperation in patients undergoing myomectomy. Combined with postoperative related indicators and follow-up results, it is found that intraoperative ultrasound monitoring is simple and does not increase operation time and hospitalization time. It is helpful for the identification and removal of hidden fibroids and can reduce the occurrence of complications, postoperative recurrence, and reoperation risks. The application of ultrasound in laparoscopic myomectomy requires the cooperation of a sonographer with a certain gynecological foundation. At the same time, the surgeon should also have a certain knowledge of ultrasound, so that the ultrasound technology can give full play to its advantages during the operation. With the development of medical technology and the continuous improvement and innovation of instruments and equipment, the application of intraoperative ultrasound in the treatment of uterine fibroids will become more and more extensive in the future, improving the safety of surgery and obtaining better clinical treatment effects. There are still some limitations in this study: first, this study is a retrospective single-center study with a small sample size and limited follow-up time; follow-up research will be explored through a large-sample, prospective, multicenter comparative trial.

## 7. Conclusion

Ultrasound monitoring can perform real-time imaging of uterine fibroids, provide the operator with important tumor location and blood supply information, and clarify the scope of tumor resection. Intraoperative ultrasound monitoring can improve the diagnostic accuracy of uterine fibroids, effectively reduce residual fibroids, completely remove small and deep fibroids, and reduce postoperative complications, recurrence, and reoperation risks, which can promote the improvement of patient prognosis effect.

## Figures and Tables

**Figure 1:** Technology roadmap.

**Figure 2:** Postoperative mean diameter of uterine fibroids.

**Figure 3:** Postoperative ultrasound examination of residual uterine fibroids in the two groups.

**Figure 4:** The recurrence of hysteromyoma by ultrasound after operation was compared between the two groups.

The article "The Influence of Intraoperative Ultrasound Monitoring on the Risk of Recurrence and Reoperation in Patients with Hysteromyomectomy" was published in 2022. Journal: Contrast Media Mol Imaging.

**Table 1:** The baseline profile.

Group	Age (years, $\bar{x}\pm s$)	Course of disease (month)	Uterine fibroid diameter (cm)	Location (cases (%))		
				Muscle intramural	Subserosal	Intermural and subserosal mixing
Research group (*n* = 40)	47.39 ± 10.93	11.05 ± 1.40	5.22 ± 1.34	32	4	4
Control group (*n* = 40)	47.62 ± 10.79	10.89 ± 1.50	5.20 ± 1.36	34	4	2
*χ* ^2^/*t*	0.120	0.493	0.066	0.727		
*P*	0.904	0.623	0.947	0.695		

**Table 2:** Comparison of surgical indicators between the two groups.

Group	Operating time (min)	The amount of bleeding during the operation (ml)	Postoperative exhaust time (h)	Hospitalization time (D)
Research group (*n* = 40)	36.02 ± 10.80	127.86 ± 35.43	26.30 ± 4.33	5.13 ± 1.12
Control group (*n* = 40)	34.70 ± 10.11	129.11 ± 35.87	27.64 ± 4.46	5.26 ± 1.18
*t*	0.564	0.157	1.363	0.505
*P*	0.574	0.876	0.176	0.614

**Table 3:** Comparison of two groups of complication rate.

Group	Cavity hematoma	Ureteral injury	Vascular nerve injury	Overall incidence (%)
Research group (*n* = 40)	1 (2.50)	1 (2.50)	0 (0.00)	2 (5.00)
Control group (*n* = 40)	4 (10.00)	3 (7.50)	2 (5.00)	9 (22.50)
*χ* ^2^				5.165
*P*				0.023

**Table 4:** The relationship between postoperative ultrasound uterine fibroids recurrence and follow-up time in two groups.

Group	Recurrence time of uterine fibroids after operation		Total recurrence rate (%)
	3∼6 months	6∼12 months	
Research group (*n* = 40)	1 (2.50)	2 (5.00)	3 (7.50)
Control group (*n* = 40)	2 (5.00)	9 (22.50)	11 (27.50)
*χ* ^2^	0.346	5.165	5.541
*P*	0.556	0.023	0.019

## Data Availability

The data used to support the findings of this study are available from the corresponding author upon request.
